The article "Combined application of zinc and silicon alleviates terminal drought stress in wheat by triggering morpho-physiological and antioxidants defense mechanisms" was retracted in 2022. Reasons: compromised peer review; a conflict of interest; concerns about the authorship.

# Combined application of zinc and silicon alleviates terminal drought stress in wheat by triggering morpho-physiological and antioxidants defense mechanisms

**DOI:** 10.1371/journal.pone.0256984

**Published:** 2021-10-07

**Authors:** Abdul Sattar, Xiukang Wang, Tahira Abbas, Ahmad Sher, Muhammad Ijaz, Sami Ul-Allah, Muhammad Irfan, Madiha Butt, Muhammad Ashfaq Wahid, Mumtaz Cheema, Sajid Fiaz, Abdul Qayyum, Mohammad Javed Ansari, Sulaiman Ali Alharbi, Milton Wainwright, Furqan Ahmad, Kui Xie, Ali Tan Kee Zuan

**Affiliations:** 1 College of Agriculture, Bahauddin Zakariya University, Layyah, Pakistan; 2 College of Life Sciences, Yan’an University, Yan’an, Shaanxi, China; 3 Department of Agronomy, Bahauddin Zakariya University Multan, Multan, Pakistan; 4 Department of Agronomy, University of Agriculture Faisalabad, Faisalabad, Pakistan; 5 School of Science and the Environment, Memorial University of Newfoundland, Corner Brook, NL, Canada; 6 Department of Plant Breeding and Genetics, The University of Haripur, Haripur, Pakistan; 7 Department of Agronomy, The University of Haripur, Haripur, Pakistan; 8 Department of Botany, Hindu College Moradabad (Mahatma Jyotiba Phule Rohilkhand University Bareilly), Bareilly, Uttar Pradesh, India; 9 Deptartment of Botany & Microbiology, College of Science, King Saud University, Riyadh, Saudi Arabia; 10 Department of Molecular Biology and Biotechnology, University of Sheffield, Sheffield, United Kingdom; 11 Institute of Plant Breeding and Biotechnology, MNS University of Agriculture Multan, Multan, Pakistan; 12 Institute of Crop Science, College of Agriculture and Biotechnology, Zhejiang University, Hangzhou, P. R. China; 13 Faculty of Agriculture, Department of Land Management, Universiti Putra Malaysia, Serdang, Selangor, Malaysia; Ghazi University, PAKISTAN

## Abstract

Wheat is an important global staple food crop; however, its productivity is severely hampered by changing climate. Erratic rain patterns cause terminal drought stress, which affect reproductive development and crop yield. This study investigates the potential and zinc (Zn) and silicon (Si) to ameliorate terminal drought stress in wheat and associated mechanisms. Two different drought stress levels, i.e., control [80% water holding capacity (WHC) was maintained] and terminal drought stress (40% WHC maintained from BBCH growth stage 49 to 83) combined with five foliar-applied Zn-Si combinations (i.e., control, water spray, 4 mM Zn, 40 mM Si, 4 mM Zn + 40 mM Si applied 7 days after the initiation of drought stress). Results revealed that application of Zn and Si improved chlorophyll and relative water contents under well-watered conditions and terminal drought stress. Foliar application of Si and Zn had significant effect on antioxidant defense mechanism, proline and soluble protein, which showed that application of Si and Zn ameliorated the effects of terminal drought stress mainly by regulating antioxidant defense mechanism, and production of proline and soluble proteins. Combined application of Zn and Si resulted in the highest improvement in growth and antioxidant defense. The application of Zn and Si improved yield and related traits, both under well-watered conditions and terminal drought stress. The highest yield and related traits were recorded for combined application of Zn and Si. For grain and biological yield differences among sole and combined Zn-Si application were statistically non-significant (*p>*0.05). In conclusion, combined application of Zn-Si ameliorated the adverse effects of terminal drought stress by improving yield through regulating antioxidant mechanism and production of proline and soluble proteins. Results provide valuable insights for further cross talk between Zn-Si regulatory pathways to enhance grain biofortification.

## Introduction

Wheat (*Triticum aestivum* L.) is one of world’s most important staple food crops. Overall, yield potential of wheat is limited due to climate change effects, especially abiotic stresses, including heat, salinity and drought [1]. Although all environmental stresses negatively affect the growth and development of wheat, terminal drought stress hampers reproductive development and grain yield [2]. In arid and semi-arid region, there is deficiency of water for wheat crop during the late season, which is considered as terminal drought that occurs at reproductive and grain-filling growth phases. Reproductive and grain-filling phases are considered as most sensitive to drought [3], and prolonged terminal drought can cause significant reduction in wheat yield [2,3]. Both, terminal drought tolerance and grain yield represent complex traits and comprehensive understandings of physiological responses under terminal drought are needed. Drought stress affects at all growth stages of wheat, and reproductive stage, particularly grain filling stage is the most sensitive where onset of drought leads to fewer and smaller grains in wheat [3]. Terminal drought stress reduces assimilate partitioning and inhibits the activities of important enzymes involved in the preparation of synthetic processes of sucrose and starch [4,5]. Drought stress disrupts nutrients relations in plant by reducing nutrients’ availability, uptake, transport and accumulation [6]. Drought induces oxidative stress due to overproduction of reactive oxygen species (ROS) [7] like hydrogen peroxide, hydroxyl radical, superoxide and singlet oxygen that can damage biological membranes through biochemical reactions [8,9]. Plants have evolved physiological (like production of osmolytes and soluble sugars) and antioxidant defense mechanisms (like ascorbate peroxidase (APX), superoxide dismutase (SOD), catalase (CAT) and peroxidase (POD) to combat the toxicity of ROS [10].

Zinc (Zn) is an important micronutrient serving as a physical, structural or regulatory cofactor for numerous enzymes [11], and regulates plants’ growth and development. Zinc supplementation reduces production of ROS and protects cells from ROS-induced damage. Zinc deficiency can lead to high ROS production and cell damage [12]. Under drought condition, Zn-deficiency became more prominent in wheat planted in Zn-deficient soil [13]. It is reported that foliar use of Zn regulated nutrients balance and stomata opening in maize to diminish the adversities of water deficit [14]. Adequate Zn fertilization significantly enhanced the activities of POD, SOD and CAT enzymes in response to water deficit [15,16]. In another study, it was documented that optimum Zn dose maintained water status, stomatal conductance and osmotic adjustment in chickpea under drought stress [17]. Moreover, Zn application improves leaf area, chlorophyll contents and other photosynthetic pigments, and stomatal conductance; thus, results in improved growth and yield [18–20]. After oxygen, silicon (Si) is the second most abundant element in soil; however, it is not as essential as other well-known inorganic nutrients. The Si, on the other hand, is a helpful nutrient that plays an essential function in plants under stress conditions [21–23]. Silicon application have been proved effective in reducing and mitigating the harmful effects of several abiotic stress on plants, including drought, salinity, heavy metals and high temperature [21,22,24]. Moreover, Si application under drought stress maintained water status of plant leaves and increased photosynthetic activity of maize crop [25]. Exogenous application of Si can make the silica-cuticle binary layer on the leaf epidermal tissue and it improved tissue water status in wheat crop [26,27].

Furthermore, both Zn [18,28] and Si [6,23] can improve anti-oxidative defense mechanisms (both enzymatic and non-enzymatic); thus, avoid damage from ROS produced by various abiotic stresses. Although individual effect of Zn or Si to alleviate abiotic stresses are well reported [18,27,29], there is lack of knowledge on the combined effect of Zn and Si to regulate physiological and biochemical mechanisms to improve grain yield of wheat under stress conditions. Therefore, major objective of this study was to investigate the potential of sole and combined application of Zn and Si to regulate physio-biochemical mechanism under terminal drought stress for sustainable wheat yield. It was hypothesized that drought stress will negatively affect the growth and physio-biochemical mechanisms of wheat under terminal drought stress, while combined application of Zn and Si will ameliorate the adverse impacts of terminal drought stress.

## Materials and methods

### Experimental site, soil and treatments

A pot experiment was conducted at College of Agriculture, Bahauddin Zakariya University, Bahadur Sub Campus Layyah, Pakistan (longitude 70° 56’ 20.5" E, latitude 30° 57’ 40.6" N, and altitude 151 m) to investigate the effect of sole and combined application Zn and Si to ameliorate the adverse effects of terminal drought stress in wheat. Two drought stress levels, i.e., control (80% water holding capacity (WHC) maintained throughout the growing season) and terminal drought stress (40% WHC maintained from BBCH growth stage 49 to 83) combined with five foliar applied Zn-Si combinations (i.e., control, water spray, 4 mM Zn, 40 mM Si, 4 mM Zn + 40 mM Si). The Zn and Si were foliar-applied 7 days after the imposition of drought stress. Seed of commercial wheat cultivar ‘Faisalabd-2008’ was obtained from Ayub Agricultural Research Institute, Faisalabad, Pakistan. The experiment was conducted in the earthen pots, each having 45 cm height and 14.5 cm diameter. The pots were filled with 15 kg of well ground air-dried sieved soil. The soil used in experiment was sandy loam (pH 8.5), electrical conductivity (EC) 2.56 dSm^-1^, organic matter 0.76%, total nitrogen 0.58 g kg^-1^, available phosphorous 9.53 mg kg^-1^ and available potassium of 62.34 mg kg^-1^. Bulk density of the soil was 1.71 g cm^-3^ and soil water content at field capacity (FC) was 20.87%. The nitrogen (N), phosphorus (P) and potassium (K) fertilizers were applied keeping the application rate of 100, 90 and 60 mg kg^-1^of soil during the time of pot filling. The sources of fertilizers were urea, di-ammonium phosphate and potassium sulphate for N, P and K, respectively. Ten uniform sized seeds were manually sown in each pot on November 15, 2019 at a depth of 3 cm. After one week of emergence three plants per pot were maintained for the subsequent studies. All pots were irrigated with tap water to maintain 80% WHC until the initiation of drought stress treatment. Two levels of soil WHC were maintained through gravimetric basis at reproductive stage of wheat.

### Data collection

#### Photosynthetic pigments and relative water contents

Keeping in view Arnon’s procedure [30], 0.5 g fresh fully expanded flag leaves were taken. At 0–4°C, 80% of 5 mL acetone was used for extraction, overnight. The supernatant was separated after centrifugation for absorbance reading at 645 and 663 nm for chlorophyll a and b, respectively by using the Spectrophotometer (Hitachi-U2001, Tokyo, Japan). Fully expanded flag leaves were used for measuring relative water contents (RWC) [31]. Selected leaves were rehydrated by bathing in deionized water for 24 hours. Fully turgid leaves were weighed and subsequently oven dried for 48 hours at 80°C.


$$RWC\;(\%)=\frac{FW-DW}{TW-DW}\times 100$$

Here; FW is fresh weight, DW is dry weight and TW is turgid weight.

#### Enzymatic antioxidants activities

Fresh leaf sample was centrifuged (15000 × g for 20 min) with 5 ml of phosphate buffer (50 mM with 7.8 pH). The inhibition of NBT (nitroblue tetrazolium) reduction provide basis for superoxide dismutase (SOD) activity estimation at 560 nm [32]. The reactants of the reaction were 1 mL NBT (50 μM), 1 mL riboflavin (1.3 μM), 50 μL enzyme extract, 950 μL phosphate buffer (50 mM), 500 μL methionine (13 mM) and 500 μL EDTA (75 mM). The exposure of reaction mixture to 30 W fluorescent lamp illuminance initiated the reaction, which was then stopped after 5min by turning off the lamp. The blue formazan formed due to NBT reduction and was observed at 560 nm. Blank reading was taken using same reactants but having no enzyme extract. Catalase activity (CAT) was recorded at 240 nm due to production of H_2_O_2_ as a result of enzyme reaction using a UV-visible spectrophotometer. To initiate the reaction, the reaction mixture (900 μL H2O2 (5.9 mM) and 2 mL phosphate buffer (50 mM) was added with 100 μL enzyme extract. The μmol of H_2_O_2_ per minute per mg of protein was used to define catalase [33]. The peroxidase (POD) activity was estimated with the protocol given by Kar and Mishra [34]. The reactants used were composed of5 ml of Tris-HCl buffer (0.1M), 5 ml pyrogallol (10 mM), 5 mM of H_2_O_2_ (5 mM) and 100 μL enzyme extract. The By noting the decline in the absorbance at 425 nm which was due to H_2_O_2_ dependent oxidation of pyrogallol, POD activity was measured as POD IU per minute per mg of the protein.

#### Determination of osmolytes

The 0.5 g healthy fresh green flag leaf sample was used for total soluble protein and free proline estimation. Pre-chilled mortar pestle with extraction buffer (pH 7) was used for sample grinding. Cocktail protease inhibitors of concentration 1 μM was added to saline phosphate buffer having 2 mM KH_2_PO_4_, 2.7 mM KCl, 10 mM Na_2_HPO_4_ and 1.37 mM NaCl dissolved in 1 L of di-ionized H_2_O before protein extraction from samples. Buffer pH was adjusted using HCl and autoclaved. Supernatant was collected after centrifugation (12000 × g for 5 min) of extracted samples and was used for measuring the quantity of soluble proteins. Bradford [35] was followed for the determination of total soluble proteins. The dilutions of10, 20, 30, 40, 50, 60, 70, 80, 90 and 100 μg μL^-1^ (Bovine serum albumin) provided basis for standard curve construction. The incubated tubes were added with 400 mL dye stock and DI water and vortexed. The absorbance was recorded using UV 4000 UV-VIS spectrophotometer. Simaei et al. [64] were followed for proline determination. Fresh leaf samples were homogenized using sulpho-salicylic acid (3% w/v) (10 mL). The filtrate was separated and kept in test tubes for color development. Then it was treated with glacial acetic acid and ninhidrine (2.5%). Afterwards these were retained in water bath whose temperature was elevated to 100°C for period of 60 min. After exclusion from water bath, toluene was added to test tubes for chromophores separation.

#### Yield and yield-related traits

At maturity, plant height and spike length of randomly selected plants from each pot was measured using standard procedure. Manually harvested and threshed plants were used to record number of grains per spike, 100-grain weight (g), biological yield and grain yield per plant (g).

### Statistical analysis

Using Fisher’s Analysis of Variance technique, all the data of the experiment was analyzed considering a two-factor complete factorial completely randomized design, and average of treatments was computed by LSD test [36]. Figures were prepared using Microsoft Excel ©365. Minimal dataset of the study used in the analysis is given in supporting information S1 Dataset.

## Results

### Photosynthetic pigments and relative water contents

Photosynthetic pigments and relative water contents (RWC) of flag leaves were reduced under drought stress (Fig 1). However, Chl a, Chl b, and Chl a+b were enhanced by foliar application of Zn and Si alone and in combination under both water availability regimes. Foliar application of Zn or Si alone and their combination enhanced Chl a content by 5.14, 1.4 and 7.3%, Chl b contents by 17.6, 7.14 and 27.5%, and Chl a+b contents by 7.5, 2.4 and 11.59%, respectively, under terminal drought stress as compared to control treatment. Foliar treatments had non-significant effect on Chl a/b contents. The Chl a content was significantly increased by foliar application of Zn, Si and their combination, and these enhanced Chl a contents by 12.5, 6.5 and 17.24%, chl b contents by 14.28, 13.04 and 20%, and Chl a+b contents by 12.93, 7.62 and 17.66%, respectively under well-watered conditions. However, other foliar treatments did not show any significant effect on Chl a/b under well-watered conditions. Overall, the highest chlorophyll contents were observed from the plants treated with combined Zn and Si under both well-watered conditions and terminal drought stress (Fig 1).

**Fig 1:** Effect of individual and combined application of Zn and Si on chlorophyll a (a), chlorophyll b (b), chlorophyll a+b (c) and relative water contents (d) of wheat under terminal drought stress. Every column in each graph represents the means (±SE) of three replicates. Zn = zinc, Si = silicon.

Relative water contents (RWC) of flag leaves of were significantly affected by foliar treatments. The RWC was enhanced by 16.38, 17.88 and 20.40% under terminal drought stress, while an increase of 0.31, 6.24 and 7.36% was recorded for Zn, Si and their combination, respectively under well-watered conditions (Fig 1).

### Activities of antioxidant enzymes

Activities of all antioxidant enzymes were significantly affected by terminal drought stress and Zn-Si application. Catalase activity was significantly increased by terminal drought stress. Foliar application of Zn and Si further enhanced catalase activity. Sole and combined application of Zn and Si enhanced the catalase activity by 25.12, 30.81 and 35.71%, respectively under terminal drought stress compared to control (Fig 2). Terminal drought stress enhanced SOD activity. Foliar application of Zn and Si further enhanced SOD activity under terminal drought stress and well-watered conditions. Sole application of Zn, Si and their combination enhanced SOD activity by 12.64, 16.54%and 18.77%, respectively under terminal drought stress compared to control. Foliar applied Zn, Si and their combination improved SOD activity by 20.24, 19.15 and 21.51%, respectively under well-watered conditions (Fig 2). Peroxide activity was increased with imposition of terminal drought stress. Foliar application of Zn, Si and Zn+Si improved peroxide activities by 23.37, 27.25 and 29.19%, respectively under terminal drought stress compared to control. While under well-watered conditions, peroxidase activity was increased by 6.5, 14.20 and 18.28% with the application of Zn, Si and Zn+Si, respectively. The highest peroxidase activity was observed for combined Zn and Si application under both water availability regimes (Fig 2). The activity of ascorbate peroxidase was increased by 31.64, 22.85 and 39.55% with foliar spray of Zn, Si and their combination, respectively under terminal drought stress. The highest activity was observed under terminal drought stress with combined application of Zn and Si (Fig 2).

**Fig 2:** Effect of individual and combined application of Zn and Si on catalase (a), superoxide dismutase (b), peroxidase (c) and ascorbate peroxidase (d) of wheat under terminal drought stress. Every column in each graph represents the mean (±SE) of three replicates. Zn = zinc, Si = silicon.

### Accumulation of osmolytes

Terminal drought stress significantly (*p<0*.*05*) affected proline content and soluble protein. However, foliar application of Zn, Si and Zn+Si increased proline and soluble proteins under terminal drought stress. Foliar applied Zn, Si and their combination enhanced proline contents by 19.15, 20.35 and 28.81%, respectively under terminal drought stress compared to control (Fig 3). The application of Zn and Si had non-significant impact on these attributes under well-watered conditions. Soluble protein contents were enhanced under terminal drought stress. Foliar application of Zn and Si alone had almost same effect on protein content and enhanced it by 19.71 and 20.33%, respectively under terminal drought stress. Nonetheless, combination of Zn and Si enhanced the protein contents by 28.81% under terminal drought stress as compared to control (Fig 3).

**Fig 3:** Effect of individual and combined application of Zn and Si on proline (a) and protein contents (b) wheat under terminal drought stress. Every column in each graph represents the mean (±SE) of three replicates. Zn = zinc, Si = silicon.

### Yield and yield-related traits

Plant height, yield and yield components, i.e., spike length, number of grains per spike, 100-grain weight, grain yield and biological yield were significantly (p<0.05) disrupted by terminal drought stress (Tables 1 and 2). Foliar application of Zn, Si and Zn+Si significantly enhanced plant height, yield and yield components under well-watered conditions and terminal drought stress. Foliar application of Zn, Si and their combination enhanced plant height by 9.15%, 9.27% and 12.10%, respectively under terminal drought stress as compared to control treatment (Table 1). The adverse effect of terminal drought stress on spike length was alleviated by foliar application of Zn and Si. Similarly, number of grains per spike was increased by 23.57, 19.78 and 27.05% with foliar application of Zn, Si and Zn+Si, respectively under terminal drought stress as compared to control treatment (Table 1). The decline in 100-grains weight was noticeably lesser where Zn and Si were foliar applied as compared to treatments without Zn and Si application. Sole application of Zn and Si improved 100-grains weight 18.71 and 14.06%, respectively, while the heaviest 100-grains were recorded with combined application of Zn and Si (Table 2). Results revealed that grain yield was significantly reduced under terminal drought stress. However, foliar application of Zn, Si and Zn+Si considerably increased grain yield by 20.93, 17.07 and 24.63%, respectively under terminal drought stress as compared to control treatment (Table 2). The negative impacts of terminal drought stress on biological yield was alleviated with foliar application of Zn and Si. Foliar-applied Zn, Si and Zn+Si improved biological yield by 23.39, 18.40 and 29.90%, respectively under terminal drought stress as compared to control treatment (Table 2).

**Table 1:** Influence of individual and combined application of zinc and silicon on plant height, spike length and number of grains per spike of wheat under drought stress conditions.

Treatments	Plant height (cm)		Spike length (cm)		Number of grains per spike	
	Well-watered	Terminal drought	Well-watered	Terminal drought	Well-watered	Terminal drought
**Ck**	83.0±2.46 cd	67.5±0.92 g	9.76±0.23 c	7.79±0.20 f	43.10±0.84 d	29.60±0.31h
**H**_**2**_ **O**	84.9±0.85 bc	69.7±1.70 fg	9.67±0.22 c	7.80±0.05 f	44.76±0.53 d	29.78±0.21h
**Zn**	90.6±2.64 ab	74.3±1.86 ef	10.31±0.23 bc	8.53±0.13 ef	48.95±0.38 c	38.73±0.41g
**Si**	89.4±4.33 ab	74.4±1.86 ef	10.80±0.33 b	8.80±0.12 e	51.48±0.19 b	36.90±0.32 f
**Zn + Si**	93.5±1.13 a	76.8±0.48 de	12.03±0.16 a	8.90±0.02 de	54.05±0.17 a	40.58±0.25 e
**LSD≤0.05**	6.51		0.84		1.75	

Each value in column of table represents the means ± SE of three replicates. Ck = control, Zn = zinc, Si = silicon, LSD = least significant difference.

**Table 2:** Influence of individual and combined application of zinc and silicon on 100-grain weight, grain and biological yield of wheat under terminal drought stress.

Treatments	100-grain weight (g)		Grain yield (g plant^-1^)		Biological yield (g plant^-1^)	
	Well-watered	Terminal drought	Well-watered	Terminal drought	Well-watered	Terminal drought
**Ck**	4.16±0.03 d	2.78±0.05 g	4.21±0.08 d	3.06±0.03 g	15.35±0.40 c	10.15±0.15 e
**H**_**2**_ **O**	4.22±0.06 d	2.82±0.04 g	4.20±0.09 d	3.07±0.06 g	15.28±0.33 c	10.28±0.08 e
**Zn**	4.89±0.03 b	3.42±0.03 f	5.04±0.04 b	3.87±0.04 ef	20.00±0.48 ab	13.25±0.42 d
**Si**	4.65±0.02 c	3.20±0.03 f	4.72±0.09 c	3.69±0.03 f	17.73±0.55 bc	12.44±0.24 de
**Zn + Si**	5.14±0.12 a	3.78±0.09 e	5.41±0.01 a	4.06±0.02 e	21.25±0.85 a	14.48±0.22 d
**LSD≤0.05**	0.22		0.29		2.92	

Each value in column of table represents the means ± SE of three replicates. Ck = control, Zn = zinc, Si = silicon, LSD = least significant difference.

## Discussion

Low water availability, especially in arid and semi-arid regions have limited wheat growth and yield performance owing to lesser nutrient availability [37,38]. The impact of drought stress on crop yield is largely determined by its severity and span, which contribute towards reduced life cycle and grain filling duration of wheat crop. In current investigation, terminal drought stress imposed negative impact on wheat growth as evidenced by reduction in photosynthetic pigments and water relations. The earlier plant response to drought is decreased relative water contents, which is reflected by reduction of leaf water potential, causing stomatal closure [39,40]. Stomatal closure reduces the transpiration rate causing an increase in leaf temperature. This high temperature leads to denaturation of membrane proteins, disturbing various biochemical mechanisms of plants, including photosynthesis, respiration, nutrient transport and assimilation, protein synthesis and enzyme activity [23,41]. Low water access to plants during their active growth period causes alterations in mineral-nutrient relations leading to poor nutrient availability and transport processes partitioning [42,43]. Plant mineral nutrient status is responsible for effective water use efficiency and helps in mitigation of stress induced negative impacts [18,42].

Zinc (Zn) and silicon (Si) are mineral nutrients which aids in improving water use efficiency of plants [44,45]. Foliar application of Zn and Si improved chlorophyll contents and leaf water contents both under terminal drought stress and well-watered conditions. Improved chlorophyll contents attributed to the role of Zn and Si in proteins and enzymes synthesis, its role as co-factor in pigment synthesis [46,47] and suppressing the activity of chlorophyll degrading enzymes (chlorophyllase) which become more active during stress conditions [48,49]. Combined application of Zn and Si stimulated photosynthetic pigment contents and relative water contents, which showed the synergistic response of both mineral nutrients. The mechanism of both nutrients supported the wheat plants under water stress, which have resulted in better growth and yield.

Water deficit conditions give rise to oxidative stress by generation of reactive oxygen species (ROS), which is counteracted by antioxidant defense mechanism of plants [50,51]. This defense mechanism involves various enzymes and non-enzymatic molecules, which convert these harmful oxygen species to water and oxygen and reduces their negative impact on plant growth [52]. Terminal drought stress increased levels of CAT, SOD, POD and APX as compared to control (no stress) in the current study. The application of Zn and Si enhanced the activity of these antioxidant enzymes under water deficit conditions, being more pronounced when applied together. Yavas and Unav [15] and Sultana et al. [19] reported enhancement in enzymatic antioxidant defense system in Zn supplemented wheat under water deficit conditions. The Zn is reported to demonstrate protective role against ROS induced damage of membranes [12,53]. The impact of applied Zn on antioxidant defense system varies with amount of Zn applied and plant growth phase, at which it is applied. The Si is well-known to enhance antioxidant enzyme activity and reduce oxidative damage under stress conditions, which confer stress tolerance capability to plants [54]. Improvement in antioxidant enzyme activity is assessed through decreased malondialdehyde contents and H_2_O_2_ contents as noted in sunflower (*Helianthus annuus*), chickpea (*Cicer arietinum*) [55,56], lentil (*Lens culinaris*) [57] and wheat leaves [58].

An enhancement in proline contents and total protein contents were recorded under terminal drought supplemented with Zn, Si and Zn + Si. The enhancement was only recognizable under stressed conditions being more prominent with Zn + Si. Proline is an important osmolyte, which is helpful in osmotic homeostasis regulation in stressed conditions [59]. The Zn has been related to amino acid synthesis, which aids in protecting plant from drought related consequences [60,61]. The compatible solute accumulation leads to improved turgor potential and water contents of plants, which contributed in improving plant growth performance under stressed condition. Silicon is also reported to stimulate compatible solute contents and protein contents under stressed conditions [62]. The compatible solute modifies plant water status and help plant to survive in stressed conditions. The combine supplementation of Zn and Si both acted synergistically with respect to proline and total protein contents.

Foliar-applied Zn and Si alone or in combination stimulated plant growth and yield parameters of wheat under terminal drought stress. It might be attributed to stimulated biochemical and physiological processes of wheat in response to applied nutrients. The protective effects of Zn and Si against ROS, membrane damage and enhancement in photosynthetic pigments, proline and total protein contents and relative water contents have improved plant growth performance. This improved growth is evident from spike length, number of grains per spike, 100-grain weight, grain and biological yield. The improvement in plant growth parameters as a result of Zn under stressed conditions attributed to the improved chlorophyll contents, antioxidant defense mechanism and production of osmolytes due to the application of Zn and Si [23,63–67].

## Conclusions

Terminal drought stress reduced the growth and productivity of wheat by reducing chlorophyll contents and production of reactive oxygen species (evident from increased antioxidant activities). The losses caused by terminal drought stress can be minimized by foliar application of Zn and Si that improves the antioxidant mechanism and production and proline and soluble proteins to regulate the plant growth under stress conditions. Based on the results, combined application of Zn and Si is suggested to ameliorate the adverse effects of terminal drought stress. However, before a wider recommendation, field trails are required under different agro-climatic conditions.

## Supporting information

S1 Dataset Minimal dataset of the study used to build tables/graphs presented in the manuscript. (XLSX)
